# The Alveolar Ridge Splitting Technique on Maxillae: A Biomechanical Human Cadaveric Investigation

**DOI:** 10.1155/2020/8894471

**Published:** 2020-11-19

**Authors:** Fabian Duttenhoefer, Peter Varga, Dominik Jenni, Leonard Grünwald, Luisa Thiemann, Boyko Gueorguiev, Andres Stricker

**Affiliations:** ^1^University Hospital of Freiburg, Germany; ^2^AO Research Institute Davos, Switzerland

## Abstract

The alveolar ridge splitting technique (ARST) offers an alternative to classic ridge augmentation techniques for successful insertion of dental implants. However, the buccal lamella is at risk of fracturing during ARST distraction. To better understand the fracture mechanisms and displacement limits of the split lamella, this study conducted biomechanical tests on human cadaveric maxilla specimens having extremely atrophied alveolar ridges treated with ARST. A total of 12 standardized alveolar splits were prepared on the maxillae of 3 elderly female donors using an oscillating piezoelectric saw. Mimicking the surgical distraction process of the lamella, each split was tested to failure using a dental osteotome attached to the crosshead of an electromechanical testing system. All specimens were scanned by means of high-resolution peripheral quantitative computed tomography prior to and post testing to evaluate split geometries and failure modes. Split stiffness, failure force, and displacement were 27.4 ± 18.7 N/mm, 12.0 ± 8.4 N, and 0.97 ± 0.31 mm, with no significant differences between anatomical sides and split locations (*p* ≥ 0.17). Stiffness correlated significantly with failure force (*R*^2^ = 0.71, *p* < 0.01). None of the alveolar split widths correlated significantly with the outcomes from biomechanical testing (*p* ≥ 0.10). The results suggest that simple geometrical measures do not predict the allowed extent of lamella distraction prior to failure. More sophisticated methods are required for surgical planning to optimize the ARST outcomes. Still, the present study may advocate a clinical protocol for the maxilla where the implant site is prepared directly after osteotomy setting and immediately before full lamella dislocation, when the lamella is still stable, resistant to mechanical stress, and bone loss caused by the abrasion of the burr is minimized.

## 1. Introduction

Rehabilitation of strongly atrophied alveolar ridge using dental implants usually requires complex augmentation techniques for their successful insertion. As an alternative to the classic augmentations through bone grafts or guided bone regeneration, the splitting and expansion of the alveolar ridge, so-called alveolar ridge splitting technique (ARST), offers the possibility of increasing the width of the alveolar ridge. This method is applied when the alveolar ridge exhibits sufficient vertical bone height but has insufficient horizontal width. After splitting and expansion of the bone, a sufficiently wide implantation site can be provided to allow full anchorage of the implant in the autologous bone [1–3]. Comparable success rates to augmentations with bone blocks or guided bone regeneration can be achieved with this technique [4]. Further ARST advantages are that a second operation is avoided and the treatment duration is shortened due to simultaneous implant insertion [5].

The technical ARST implementation consists of setting a longitudinal osteotomy along the course of the alveolar ridge at the location of planned implant insertion and two vertical relief osteotomies. The enlarged alveolar width is then created by careful distraction of the outlined buccal segment [6, 7]. Subsequently, a drilling protocol is applied, and the implant is inserted.

The main risk of this surgical technique is related to fracturing of the buccal lamella during distraction. The risk increases significantly in case of advanced alveolar ridge atrophy due to high bone resorption and poor bone quality [4, 8–14]. So far, little scientific knowledge exists about the fracture mechanisms and maximum possible extent of distraction before a lamella fracture occurs. Previous work investigated lamellar fracturing in porcine specimens [15]. Another in vitro animal study developed a biomechanical model to simulate the surgical procedure and fracture behavior during alveolar bone splitting [16]. However, both those previous investigations were limited by the use of porcine specimens which may differ from the human tissue. In particular, the good animal bone quality did not necessarily represent a situation with the most endangered patients, being the targeted group with atrophic alveolar ridge. Therefore, ARST and in particular the phenomenon of lamellar fracturing should be investigated on relevant human bone tissue.

The aim of this study was to perform biomechanical testing on human cadaveric specimens representing patients at the highest risk of lamellar fracturing during ARST implementation in order to investigate better the maximum extent of lamella displacement, draw conclusions about the predictability, and ultimately help prevent intraoperative lamellar fractures.

## 2. Materials and Methods

### 2.1. Specimen Preparation and Scanning

Fresh-frozen (-20°C) human cadaveric heads of three elderly female donors (76, 83, and 89 years old) with a long-standing complete edentulous intraoral condition were used. The donors gave their informed consent inherent within the donation of the anatomical gift statement during their lifetime. The maxillae were dissected from the skulls by Le Fort I osteotomy using an oscillating surgical saw (DePuy Synthes, Oberdorf, Switzerland), then separated and cleaned of soft tissues. Alveolar splits of 8 mm depth and 10 mm width were prepared using an oscillating piezoelectric saw with a blade thickness of 0.35 mm in two maxillae and 0.55 mm in the third one (PIEZOSURGERY® touch, Mectron, Carasco, Italia) (Figure 1). Vertical relief incisions were performed at both ends perpendicularly to the split plane. Twelve splits were prepared in total—four per maxilla: one in the canine and one in the premolar region of its left and right sides (Figure 1).

All prepared specimens were scanned by means of high-resolution peripheral quantitative computed tomography (HR-pQCT, XtremeCT, Scanco Medical AG, Brütisellen, Switzerland) to investigate the osteotomy lines. Scanning settings were 60 kV voltage, 900 *μ*A current, and 82 *μ*m isotropic voxel size. The dimensions of the alveolar bone were measured on the postoperative HR-pQCT images using Amira software package (Version 6.0, FEI, Hillsboro, USA) including the crestal and basal widths on the buccal and oral sides of the split, as well as the total crestal and basal widths (Figure 2).

### 2.2. Biomechanical Testing

The specimens were positioned in a custom-made adjustable holder. The cranial aspect of the maxillae was embedded in dental cement (True-Plast, Superhartgips, Benzer Dental AG, Zurich, Switzerland) that cured at room temperature for approximately one hour. The embedding level was sufficiently far away from the splits in order to avoid its influence on the alveolar split behavior during the subsequent biomechanical tests (Figure 3, left).

Each split was tested to failure in a setup mimicking the surgical expansion process as follows. First, the plane of the split, identified by a thin plate inserted in the osteotomy, was carefully aligned with the horizontal plane by rotating the ball joint of the adjustable specimen holder (Figure 3, left). The aligned specimen was then mounted on an electromechanical material testing machine (Instron 5866, Instron, Norwood, USA). A dental osteotome (Ergoplant, Aesculap AG, Tuttlingen, Germany) was attached to a 1 kN load-cell mounted on the crosshead of the testing machine. The osteotome blade was aligned horizontally, and its height was adjusted to the split plane. The osteotome blade was then carefully inserted into the split at 3 mm depth by moving the specimen holder along the osteotome axis. The position of the specimen holder was then fixed. Quasi-static distraction test of the buccal lamella was performed by displacement-controlled vertical translation of the osteotome at a rate of 5 mm/min in vertical (i.e., vestibular) direction along the machine axis (Figure 3, right).

All specimens were rescanned post testing by means of HR-pQCT using the same settings as described above. Surface mesh of the segmented bone image region was used to visualize the fracture lines in Amira.

### 2.3. Data Acquisition and Analysis

Displacement of the machine crosshead and reaction force was recorded by the controllers of the testing system at a rate of 10 Hz. Stiffness (*K*, in N/mm) was evaluated from the steepest slope in the linear portion of the force-displacement curve. Failure was defined by a significant drop in the reaction force during testing. The corresponding failure force (*F*_fx_, in N) and failure displacement (*u*_fx_, in mm) were quantified.

### 2.4. Statistical Evaluation

Normality of data distribution among all geometrical alveolar widths and biomechanical outcomes was screened using the Shapiro-Wilk test. Friedman and Wilcoxon Signed-Rank tests were applied to detect significant differences among alveolar widths, as well as among biomechanical outcomes with respect to donors, anatomical sides, and anatomical locations. Spearman test was used to identify significant correlations between alveolar widths and biomechanical outcomes. Level of significance was set to *p* = 0.05 for all statistical tests.

## 3. Results

The measured alveolar widths of all prepared specimens (crestal-buccal, crestal-oral, crestal-total, basal-buccal, basal-oral, and basal-total) are summarized in Table 1. The dimensions of the splits were more standardized on the buccal side of the split and showed a larger scatter on the oral side. Overall, these geometrical parameters were significantly different for donor A compared with both donors B and C (*p* ≤ 0.03) and did not differ significantly between donors B and C (*p* = 0.22). No significant differences in the corresponding alveolar widths were detected between donors' right and left sides (*p* = 0.11). Moreover, the canine alveolar widths of the donors did not differ significantly from the corresponding premolar ones (*p* ≥ 0.34).

A typical force-displacement curve of a biomechanically tested specimen is shown in Figure 4.

All biomechanical tests resulted in clinically relevant fracture modes with levels of the fracture lines ranging between the tip of the osteotome and the basal base of the splits (Figure 5).

The outcomes from biomechanical testing (stiffness, failure force, and failure displacement) are presented in Table 1. They differed significantly for donor B compared with both donors A and C (*p* < 0.01) but did not differ significantly between donors A and C (*p* = 0.31). No significant differences in these outcomes were detected between donors' right and left sides (*p* ≥ 0.17). Moreover, the outcomes for canine anatomical location did not differ significantly from the corresponding ones for premolar location (*p* ≥ 0.36).

No significant correlations were detected between any of the measured alveolar widths and any of the outcomes from biomechanical testing (*p* ≥ 0.10). Stiffness of the tested specimens correlated significantly with their failure force (*p* < 0.01, *R*^2^ = 0.71, Figure 6), but not with the failure displacement (*p* ≥ 0.21). No significant correlation was identified between failure force and failure displacement (*p* ≥ 0.10).

## 4. Discussion

The most common complication of ARST is the intraoperative fracture of the buccal lamella [16]. It is therefore of essential importance to preoperatively estimate the maximum possible displacement of the lamella in order to adapt the surgical protocol accordingly. Still, the extension behavior of the buccal lamella and the related fracture mechanisms are not deciphered yet.

A pilot study by Stricker et al. successfully developed a biomechanical setup for relevant replication of lamellar fracturing applying ARST on porcine jaw specimens; a mean critical lamella displacement of 1.27 mm was reported for porcine mandibles osteotomized via piezosurgery and tested in lateral distraction with an osteotome [16]. Comparable results in alveolar ridge splitting of porcine mandibles were obtained in a study by Jung et al. [15] who analyzed lamella displacement by vertical force application utilizing either a mallet and chisel (control group) or an engine-driven ridge spreader (test group). The alveolar crest width could be significantly increased in both control (1.23 ± 0.45 mm) and test groups (0.98 ± 0.41 mm) [15]. Although the porcine model exhibits a close similarity to human bone in terms of structure and bone mineral density [17, 18], the model has limited relevance for alveolar ridge splitting due to the pig anatomy [15, 16]. Moreover, the pristine bone of the applied pig models does not reproduce the clinical situation of severely atrophied and brittle human alveolar ridges. It is noteworthy to mention that the lack of cancellous bone often accounts for lamellar fractures, especially in the thicker and more mineralized cortical bone, such as the one seen in the mandible [19].

In the present work, the mechanical fracture simulation was transferred to human anatomy with strongly atrophied maxillae and was therefore able to reproduce a real clinical situation in the most endangered patients' group. We focused on the maxilla as the mandible in humans is less suited for alveolar ridge splitting due to its centrifugal atrophy pattern and a rather round-shaped cross-section as compared to the wedge-shaped pattern of the maxilla seen in the classification proposed by Cawood and Howell [20]. Moreover, implant placement in the atrophied maxilla aims to place the implant as far as buccally as possible. Due to the centripetal atrophy pattern of the maxilla, alveolar ridge splitting with distraction of the buccal ridge aspect facilitates compensation of the centripetal bone loss.

In our previous porcine model, the osteotomy outlines varied between 4 and 8 mm depth being with a crestal cut between 7 and 10 mm in the mesiodistal direction [16]. The achieved displacement before permanent lamella dislocation, i.e., prior to reaching fracturing force, was 1.3 ± 0.9 mm. This considerable variation in the test results was probably related to the nonstandardized lamellar geometries. While relief height was found to correlate with fracture force, no correlations were found fracture displacement and the latter. Due to the small sample size, it could not be clearly concluded whether the scatter in the displacement results was related to the height, width, and/or the thickness of the lamella, the latter proportionally increasing with the height due to the porcine anatomy. Hence, the split geometry in the present human cadaveric study was standardized to 8 mm depth and 10 mm width. Interestingly, although the utilized human specimens showed severe alveolar ridge atrophy, the average displacement when reaching fracturing force (0.97 mm) was close to the one reported in the porcine study (1.3 mm). Nevertheless, this may have been a coincidence. In turn, the standard deviation of the results could be efficiently reduced via the aforementioned standardization. In addition, the standardized depth and width of the splits allowed to investigate whether the lamellar thickness at the basal or crestal aspect would predict the biomechanical outcomes. No significant correlations were detected between the geometrical alveolar widths and the outcomes from biomechanical testing. However, similarly to a previous animal study, it could be shown that the stiffness correlated strongly with the failure force [16]. Nevertheless, the fracture line was not always located at the base, but often more crestal, assumedly at the local weakest region of the lamella (Figure 5). These findings suggest that simple geometrical measures may not suffice, and more sophisticated methods are necessary to preoperatively predict the biomechanical outcomes and especially the clinically relevant allowed extent of lamellar distraction. Finite element analysis, successfully applied on a small set of porcine specimens in our previous study [16], appears to be a promising technique for prediction of the biomechanical behavior and fracturing of the lamella. Future research is required to evaluate whether finite element models can better predict lamellar dislocation and possible implant placement in human alveolar bone based on computed tomography scans.

During the measurements performed in the present study, in agreement with previous work [16], the maximum force of the force-displacement curve was defined as failure force. However, this may not always correspond to what is described as “fracture of the lamella” in a clinical context. In a clinical situation, the term “fracture of the lamella” usually refers to a fully detached lamella or extensive dislocation inhibiting implantation. The definition used in this study implies that, beyond the state with maximum force, no further increase in the force is measured following increase of the applied displacement; however, the lamella could still be in place attached to the base, not extensively displaced and continuing to resist to further distraction. It remains unclear whether an implant could be inserted in a split at this state. To get further insight into the bone split technique, future studies may focus on fracture mechanisms and the clinical relevance of dislocating the alveolar lamella beyond the state defined by the maximum force in this study.

Yet, we have found some evidence that may lead to improvement of the surgical alveolar bone split protocol. Most of the clinical fractures of the bone split occur during instrumentation of the lamella, especially when using rotation burrs to prepare the implant site. According to our results, we propose to prepare the implant site after osteotomizing while the lamella is slightly dislocated right to the point prior to fracturing. The latter can be feasibly controlled by removing the utilized osteotome or chisel. At this point, the lamella is still stable and resistant to mechanical stress, with preformed gap and minimal bone loss caused by the abrasion of the burr.

### 4.1. Limitations

The limitations of the study are similar to those inherent for all biomechanical cadaveric investigations using a limited number of specimens. The sample size was modest, which was mainly due to restricted availability of relevant human cadaveric material. In addition, the lamellar displacement measured by the testing system may not have been accurate enough due to certain compliance of the experimental setup. Furthermore, the biomechanical in vitro testing approach may not have perfectly mimicked the split expansion during surgery. Finally, only ridge splitting with expansion was performed in the maxilla and without implantation that might have had further effects on the stability of the lamella.

### 4.2. Conclusions

The results from the current study suggest a clinical protocol during alveolar ridge splitting in highly atrophic maxila, where the implant site can be minimal and adequately prepared directly after osteotomy setting and immediately before full lamella dislocation−identified by the maximum force before fracturing. In this state, the lamella is still stable and resistant to mechanical stress, while bone loss caused by the abrasion of the burr is minimal. More sophisticated methods are required for surgical planning to optimize the ARST outcomes, since simple geometrical measures do not predict the allowed extent of distraction prior to failure.

## Figures and Tables

**Figure 1:** Surgical procedure: maxilla with deflected soft tissue (a); horizontal osteotomies created with the alveolar ridge splitting procedure (b); preparation of alveolar splits using an oscillating piezoelectric saw (c); controlling alveolar splits dimensions of 10 mm horizontal width (d) and 8 mm vertical depth (e) following the procedure.

**Figure 2:** Geometrical measurements to quantify alveolar widths (crestal-buccal, crestal-oral, crestal-total, basal-buccal, basal-oral, and basal-total) on the high-resolution peripheral quantitative computed tomography images.

**Figure 3:** Setup for distraction testing of a split lamella. Photograph of an embedded specimen with a thin metal plate inserted in the split to identify the direction of positioning for biomechanical testing (left). Schematic illustration of the experimental setup (right).

**Figure 4:** Exemplary force-displacement curve of a specimen during biomechanical testing, with a circle indicating fracturing.

**Figure 5:** Exemplified fracture lines of alveolar split lamellae visualized on the surface renderings of segmented post-test high-resolution peripheral quantitative computed tomography images and highlighted with red ellipses.

**Figure 6:** Linear regression plot between stiffness and failure force, visualizing a significant correlation between these two outcomes from biomechanical testing (*p* < 0.01).

**Table 1:** Measured alveolar widths of all prepared specimens (crestal-buccal, crestal-oral, crestal-total, basal-buccal, basal-oral, and basal-total) together with the outcomes from their biomechanical testing (stiffness, failure force, and failure displacement).

Specimen				Alveolar width						Outcomes biomechanical testing		
Donor ID	Split ID	Side	Anatomical location	Crestal-buccal	Crestal-oral	Crestal-total	Basal-buccal	Basal-oral	Basal-total	Stiffness (*K*)	Failure force (*F*_fx_)	Failure displacement (*U*_fx_)
				[mm]	[mm]	[mm]	[mm]	[mm]	[mm]	[N/mm]	[N]	[mm]
A	1	L	Canine	1.36	0.67	2.38	2.47	0.70	3.52	60.9	34.8	0.88
A	2	L	Premolar	0.71	1.23	2.29	3.40	4.13	7.88	16.3	9.2	0.93
A	3	R	Premolar	0.88	0.82	2.05	1.90	2.51	4.76	42.1	14.9	0.9
A	4	R	Canine	0.96	0.87	2.18	1.16	2.16	4.12	31.2	15.7	0.93
B	1	L	Canine	1.02	0.86	2.43	1.50	1.56	3.61	11.4	8.6	1.27
B	2	L	Premolar	1.37	2.32	4.24	2.37	3.99	6.91	15	8.5	0.77
B	3	R	Premolar	1.22	2.22	3.99	1.99	3.05	5.59	23.1	5.1	0.5
B	4	R	Canine	1.15	1.00	2.70	1.75	2.68	4.98	5.4	4.6	1.18
C	1	L	Canine	1.05	0.70	2.10	3.50	6.55	10.40	24.2	9.8	0.59
C	2	L	Premolar	1.94	0.59	2.88	2.55	4.16	7.06	62.4	18.3	1.58
C	3	R	Premolar	0.99	0.43	1.77	2.27	3.32	5.94	23.9	6.6	0.77
C	4	R	Canine	1.03	1.13	2.51	2.90	7.15	10.41	13.3	7.6	1.3

Mean				1.14	1.07	2.63	2.31	3.50	6.27	28.7	12.0	0.97
Standard deviation				0.31	0.60	0.76	0.71	1.88	2.37	19.0	8.4	0.31

## Data Availability

The data of the submitted paper is available upon e-mail request to the corresponding author.
